# Changes in the electron paramagnetic resonance spectra of albumin-associated spin-labeled stearic acid as a diagnostic parameter of colorectal cancer

This article has been retracted.

**DOI:** 10.1186/1477-7819-11-223

**Published:** 2013-09-11

**Authors:** Zhongchao Liu, Wenyi Zhang, Saijun Fan, Liang Wang, Ling Jiao

**Affiliations:** 1 Department of Radiation Protection Center, Institute of Radiation Medicine, Chinese Academy of Medical Sciences&Peking Union Medical College, Tianjin Key Laboratory of Molecular Nuclear Medicine, 238 Baidi Road, Nankai District, Tianjin 300192, P.R. China

**Keywords:** Colorectal cancer, Discriminant analysis, EPR/ESR, Spin probe

## Abstract

**Background:**

With more than 940,000 new colorectal cancer cases worldwide each year, there is no better way for colorectal cancer routine screening. The aim of this study was to investigate whether the fatty acid binding to albumin is detectably and significantly altered in colorectal cancer patients when compared with healthy people, in order to find a better way for colorectal cancer diagnosis.

**Methods:**

One hundred and forty-one patients operatively treated for colorectal cancer were included in the examination, and 180 healthy people were also enrolled as controls. Commercial 16-doxyl stearic acid was used as spin probe. Serum albumin was analyzed by electron paramagnetic resonance (EPR) with spin probe. Discriminant analysis was carried out using the measured EPR spectra by SPSS 20.0.

**Results:**

Of the original grouped cases, 89.4% were correctly classified. Of the cross-validated grouped cases, 86.9% were correctly classified. Using Fisher linear discriminant analysis we were able to develop a mathematical model allowing for identification of colorectal cancer patients based on five values (both relative intensity and peak width) which are obtained from the EPR spectrum.

**Conclusions:**

Cancer-associated alterations to albumin can be assessed by spin-label EPR. The potential applications for this diagnostic technique are significant and represent a cost-effective means for screening patients with cancer. Spin probe for diagnosis of colorectal cancer might be a useful tool and further studies should take place in order to investigate all stages of colorectal cancer patients.

## Background

Colorectal cancer is the second most common cancer and the second most common cause of death by cancer [1]. The clinical stage of the disease at diagnosis often determines the prognosis and survival rate of a patient with colorectal cancer [2]. If the colorectal cancer patient could be diagnosed at an early stage, they will have a better treatment than if diagnosed at an advanced stage. However, insufficient evidence concerning prognostic and predictive value exists for other molecular factors such as thymidylate synthase, microsatellite instability (MSI), p-53 and K-ras. [3].

Human serum albumin (HSA) is the main component for transport of a variety of peptides and of water-insoluble fatty acids (FA) in the serum [4]. Its remarkable ability for binding FA has motivated our group to use spin-labeled derivatives of stearic acids to monitor conformational changes around its binding sites [5]. Seven long-chain FA binding sites have been described so far [6]. Proteins released from tumor cells are able to bind to albumin and thus lead to a modification of its structure and function [6,7]. As a consequence, the binding and transport capacities for FA are also changed. These changes can be detected by electron paramagnetic resonance (EPR)/electron spin resonance spectroscopy [8,9]. EPR is suitable for the determination of functional characteristics of plasma proteins [7,10]. EPR spectroscopy detects radicals that are, in the case of HSA, introduced artificially using long-chain FA that have a stable radical (doxyl) chemically attached and by analyzing how these spin-labeled FA bind to albumin [7]. Use of this technique with 16-doxyl stearic acid (2-(14-carboxytetradecyl)-2-ethyl-4, 4-dimethyl-3-oxazolidinyloxy) as spin probe has previously demonstrated cancer-specific alterations in albumin conformation [10,11]. We used EPR spectroscopy to investigate the diagnostic utility of serum albumin conformation analysis in patients with colorectal cancer and chronic disease.

## Methods

### Samples

All patients who presented to department of surgical oncology PLA People's Liberation Army General Hospital had been pathologically diagnosed with colorectal cancer during the study period. Samples were collected from 141 patients with colorectal cancer and 180 blood donors and other volunteers known to be in good health. All patients provided their consent for participation in the study (approved by Institute of Radiation Medicine Chinese Academic of Medical Sciences ethics committee). Table 1 shows the detailed information. Blood was obtained by standard venipuncture techniques and collected without any additive. After clotting, serum was separated by centrifugation for 10 minutes, isolated, and then stored at −20 °C before analysis.

**Table 1:** Demographic information for patients evaluated in the study

**Group**	**Median age (years)**	**Age range**	**Female (%)**
**I**	**72**	**40-92**	**62**
**II**	**53**	**27-87**	**46**

Group I, patients with colorectal cancer just after operation (n = 141); Group II, healthy volunteers (n = 180).

### Sample preparation

Commercial 16-doxyl stearic acid (Sigma-Aldrich GmbH, Munich, Germany) was used as spin probe. This compound was chosen because of the extremely high binding constant of albumin for stearic acid (6.9 × 10^7^ L/mol), generally leading to 99.9% binding of this spin probe to albumin. Here we used a defined concentration of spin probe-pure ethanol compounds to perform the experiment. Each aliquot received a defined concentration of spin probe-pure ethanol compounds with 50 μL of serum and then transformed to a microliter shaker for 10 minutes at 25°C covered by parafilm. The aliquots were then transferred into capillary glass tubes for analysis within the EPR spectrometer. Each sample was measured three times.

### Sample measurement

We measured the EPR spectra of each sample with a commercially available EPR spectrometer (Bruker EMX A300, Ettlingen, Germany). The spectrometer operating conditions adopted during the experiments are given in Table 2.

**Table 2:** The spectrometer operating conditions adopted during the experiment

**Central field**	**3515 G**
**Sweep width**	**150 G**
**Microwave frequency**	**9.864 GHz**
**Microwave power**	**15.94 MW**
**Modulation frequency**	**100 KHz**
**Modulation amplitude**	**10 G**
**Receiver gain**	**20**
**Sweep time**	**20 s**
**Time constant**	**0.16 ms**

As the EPR spectrum is comprised of 1024 data points, we just used Matlab (version 7.0 Math Works Natick, Massachusetts, U.S.A.) to make up a small program to simulate the spectrum curve using least-square fitting and calculated the peak width and the relative intensity.

### Statistical analysis

Gammerman and colleagues [12] and de Noo and colleagues [13] described a double cross-validatory implementation of linear discriminant analysis for the calibration of a diagnostic rule based on a single spectrum per patient (and for a single fractionation). Due to non-normal distribution of the raw data, a logarithmic transformation was needed. To permit comparisons with other studies, results are presented as means with the standard deviation obtained after the Ln transformation. Comparisons or correlations were evaluated by using non-parametric tests (Kruskall Wallis one-way variance analysis or Spearman Rank test, respectively) on the raw data, and by means of Student’s *t* test on normalized data. Discriminant analysis was carried out using the measured EPR spectra by SPSS 20.0 (IBM, Armonk, New York, U.S.A). Selected values for variables such as relative intensity and peak widths can then be used to estimate the biophysical characteristics of the 16-doxyl stearic acid spin label. The selected parameters are shown in Figure 1. The analysis was performed using the option of the 'equal prior probability' to assign the subjects to groups.

**Figure 1:** **Selected values in a typical spectrum.** ΔH1ΔH2ΔH3 show the relative intensity; ΔH4ΔH5 show the relative peak widths.

All the predictor variables were subjected to stepwise discriminant function analysis, which has the potential to optimally separate the two groups; furthermore, the statistical significance was assessed using Wilks’ lambda. The variables having the higher discriminant function coefficient were included in the discriminant function for developing the formula.

$$F=d_{i1}V_{1}+d_{i2}V_{2}+d_{\mathrm{iP}}V_{P}+C$$

Where F is the discriminant function score, d_i_ is the discriminant function coefficient, V is the score of the predictor variable and C is the discriminant function constant.

## Results

As shown in Table 3, the five selected values (shown in Figure 1) were statistically different between the two groups. The *P* values of the five parameters were all less than 0.001, which means they are significantly different between groups. Linear discriminant analysis was used based on the five selected parameters.

**Table 3:** Medians and standard deviation of the variables analyzed and means and standard deviations of Ln-transformed levels of selected values

**a)**		**ΔH1**	**ΔH2**	**ΔH3**	**ΔH4**	**ΔH5**
**Group I**	**Median**	**118244**	**122952**	**56825**	**15.3**	**15.378**
**(n = 141)**	**SD**	**24751**	**14729**	**25265**	**0.078**	**0.114**
**Group II**	**Median**	**64398**	**71980**	**43411**	**15.192**	**15.362**
**(n = 180)**	**SD**	**11498**	**12072**	**6379**	**0.051**	**0.086**
***P *value**		**<0.001**	**<0.001**	**<0.001**	**<0.001**	**<0.001**
**b)**		**LnΔH1**	**LnΔH2**	**LnΔH3**	**LnΔH4**	**LnΔH5**
**Group I**	**Median**	**11.657**	**11.697**	**10.913**	**2.728**	**2.73**
**(n = 141)**	**SD**	**0.223**	**0.219**	**0.266**	**0.007**	**0.005**
**Group II**	**Median**	**11.17**	**11.056**	**10.668**	**2.721**	**2.732**
**(n = 180)**	**SD**	**0.17**	**0.186**	**0.149**	**0.003**	**0.006**
***P *value**		**<0.001**	**<0.001**	**<0.001**	**<0.001**	**<0.001**

Group I, patients with chronic disease just after operation (n = 142); Group II, healthy volunteers (n = 180); *SD* standard deviation.

a) is the original data.

b) is the data after Ln-transformation. Ln is Logarithmic transformation. ΔH1 is changed into LnΔH1 after Ln Logarithmic transformation.

Table 4 shows the accuracy of the discriminant function coefficient for all the predictor variables which were included in the study, from which the highest accurate values were included for the generation of discriminant function. The discriminant analysis produced the best discriminant functions and the predictor variables included in the functions were ΔH1ΔH2ΔH3ΔH4 and ΔH5 based on the greatest univariate discriminant coefficient. Before the formula was calculated with the greatest univariate discriminant coefficient, they were subjected to a test of significance using Wilks’ lambda. It was found the entire assigned predictor variables showed statistical significance at *P* < 0.05 (Table 4).

**Table 4:** Wilk’s lambda to test the significance among the predictor variables

**Test of function(s)**	**Wilks’ lambda**	**Chi-square**	**Degrees of freedom**	**Significance**
**1**	**0.200**	**509.437**	**5**	**0.002**

The Fisher’s discriminant functions were as follows:

F1=338.904ΔH1+88328.145ΔH2−103.109ΔH3+96423.334ΔH4+265.178ΔH5−255051.924

F2=328.375ΔH1+88226.653ΔH2−116.781ΔH3+96324.452ΔH4+259.369ΔH5−254166.845

The value obtained using discriminant function for cancer patients and healthy people is calculated, respectively. This shows that this discriminant function formula can accurately identify cancer in this population. To access whether it is possible to generate accurate cancer diagnosis models from data collected for this study, discriminant functions were calculated and tested using cross-validation. This was performed using SPSS, and the leave-one-out method was chosen to calculate the cross-validation error rate (Table 5). The discriminant function used in the present study describes the optimal separation between the patients and healthy controls, and also shows that there are significant differences between them. This is substantiated by the classification accuracy of functions provided in Table 5. Hence, the original grouped cases correctly classified were 89.4%.

**Table 5:** Classification accuracy checked using cross-validation for the developed discriminant function

**Classification results**^**a,b**^					
		**Group**	**Predicted group membership**		**Total**
			**1**	**2**	
**Original**	**Count**	**1**	**128**	**13**	**141**
		**2**	**21**	**159**	**180**
	**%**	**1**	**90.8**	**9.2**	**100.0**
		**2**	**11.7**	**88.3**	**100.0**
**Cross-validated**^**c**^	**Count**	**1**	**124**	**17**	**141**
		**2**	**25**	**155**	**180**
	**%**	**1**	**87.9**	**12.1**	**100.0**
		**2**	**13.9**	**86.1**	**100.0**

^a^89.4% of original grouped cases were correctly classified; ^b^86.9% of cross-validated grouped cases correctly classified; ^c^cross-validation is done only for those cases in the analysis. In cross-validation, each case is classified by the functions derived from all cases other than that case.

## Discussion

Albumin is the single most abundant protein in nonpathogenic plasma, comprising approximately two-thirds of total plasma proteins [4,9,11]. This study shows that the ability of albumin to bind FA is significantly altered in patients with colorectal cancer. This modification is likely caused by the presence of bioactive peptides and other substances from tumor tissue [5,12,14]. The shape of the EPR spectrum reflects the state of the spin probe molecules, such as characteristics of its molecular motion and electrical and magnetic fields in the surrounding environment [11,15,16]. Results of recent application of EPR spectroscopy in animal models and humans suggest that EPR has great diagnostic potential [9-11].

Discriminant functions have become a widely used method for disease discrimination [12]. Stepwise discriminant function analysis was applied which calculates the optimum combination of variables for discriminant function and weighs them to reflect their contribution to the determination [12,13]. A deficiency of the current study was the significant difference in physical conditions between healthy individuals and patients with colorectal cancer. Postoperative patients only represent part of the patients with colorectal cancer. The effect of chemotherapy, which might have significant influence on tumor-related metabolite binding to albumin [15,17], as well as EPR spectral differences caused by tumor stage and localization [18,19], have not been analyzed here. Automation of the pipetting and dilution steps would also probably enhance the precision of the procedure [11].

## Conclusions

The obtained results show that cancer-associated alterations to albumin can be assessed by spin-label EPR [9,11]. Using Fisher linear discriminant analysis we were able to develop a mathematical model allowing for identification of colorectal cancer patients with an 89.4% success rate based on fives values (of both relative intensity and peak width) which are obtained from the EPR spectrum. The potential applications for this diagnostic technique are significant and represent a cost-effective means for screening patients with cancer [11,19]. Further studies should take place in order to investigate all stages of colorectal cancer patients.

### Statement

The study was approved by the local ethical committee and all individuals provided written informed consent for study participation.

## Abbreviations

EPR: Electron paramagnetic resonance; FA: Fatty acids; HSA: Human serum albumin.

## Competing interests

The authors declare that they have no competing interests.

## Authors' contributions

ZL, WZ, SF and LJ designed the study. ZL and LW carried out the study and interpreted the results. ZL wrote the manuscript. All authors read and approved the final manuscript.
